# Hydrogenolysis of Polyethylene and Polypropylene into Propane over Cobalt-Based Catalysts

This article has been retracted.

**DOI:** 10.1021/jacsau.2c00402

**Published:** 2022-10-05

**Authors:** Guido Zichittella, Amani M. Ebrahim, Jie Zhu, Anna E. Brenner, Griffin Drake, Gregg T. Beckham, Simon R. Bare, Julie E. Rorrer, Yuriy Román-Leshkov

**Affiliations:** † Department of Chemical Engineering, Massachusetts Institute of Technology, Cambridge, Massachusetts 02139, United States; ‡ SLAC National Accelerator Laboratory, Menlo Park, California 94025, United States; § Renewable Resources and Enabling Sciences Center, National Renewable Energy Laboratory, Golden, Colorado 80401, United States; ∥ BOTTLE Consortium, Golden, Colorado 80401, United States

**Keywords:** polyolefin waste, chemical recycling, cobalt, ZSM-5, propane, plastic circularity, selective hydrogenolysis

## Abstract

The development of technologies to recycle polyethylene (PE) and polypropylene (PP), globally the two most produced polymers, is critical to increase plastic circularity. Here, we show that 5 wt % cobalt supported on ZSM-5 zeolite catalyzes the solvent-free hydrogenolysis of PE and PP into propane with weight-based selectivity in the gas phase over 80 wt % after 20 h at 523 K and 40 bar H_2_. This catalyst significantly reduces the formation of undesired CH_4_ (≤5 wt %), a product which is favored when using bulk cobalt oxide or cobalt nanoparticles supported on other carriers (selectivity ≤95 wt %). The superior performance of Co/ZSM-5 is attributed to the stabilization of dispersed oxidic cobalt nanoparticles by the zeolite support, preventing further reduction to metallic species that appear to catalyze CH_4_ generation. While ZSM-5 is also active for propane formation at 523 K, the presence of Co promotes stability and selectivity. After optimizing the metal loading, it was demonstrated that 10 wt % Co/ZSM-5 can selectively catalyze the hydrogenolysis of low-density PE (LDPE), mixtures of LDPE and PP, as well as postconsumer PE, showcasing the effectiveness of this technology to upcycle realistic plastic waste. Cobalt supported on zeolites FAU, MOR, and BEA were also effective catalysts for C_2_–C_4_ hydrocarbon formation and revealed that the framework topology provides a handle to tune gas-phase selectivity.

Plastic waste represents one of the most pressing problems of modern society, as over 5000 million tonnes have been landfilled or leaked into the environment since the 1950s.^1−4^ Polyethylene (PE) and polypropylene (PP), the two most produced plastics worldwide, account for over half of this waste by weight.^1,3^ While mechanical recycling can process only a fraction of plastic waste, chemical recycling could convert it into processable products that can be reintegrated into a circular polymer economy.^5−9^ However, a key challenge lies in activating the strong and inert C–C bonds of the PE and PP backbones.

Among the different strategies reported to this end, hydrogenolysis,^9−18^ which utilizes H_2_ to cleave the polymer into shorter alkanes, is a promising approach to deconstruct PE and PP under moderate conditions. Notably, platinum- and ruthenium-based catalysts have been shown to convert model polymers and postconsumer polyolefin plastics into liquid alkanes (C_7_–C_20+_).^19−28^ To date, these catalytic systems often require high loadings of precious metals (up to 6 wt %) and typically produce a wide array of products ranging from CH_4_ and other light alkanes to liquid paraffins (C_7_–C_24_) and solid waxes (C_25+_), which stems from the internal C–C bond cleavage mechanism favored in these systems.^20−24^ The development of catalysts that are not based on precious metals and that promote narrower product distributions would enable more efficient technologies to valorize plastic waste. This would require catalysts adept at selectively cleaving the C–C bond positions in the polyolefin chain that are nonterminal, thus minimizing generation of undesired CH_4_, but near the chain end, forming a limited range of hydrocarbons, such as ethane, propane, and butane. These could be readily converted into the corresponding olefins and H_2_ by commercial, scalable dehydrogenation technologies,^29−31^ thereby regenerating the monomers and closing both the carbon and hydrogen loop in PE and PP production (Figure 1).

**Figure 1:** Simplified scheme of the envisioned closed-loop polyolefin cycle. This involves catalytic hydrogenolysis of waste plastic at close-to-terminal C–C bonds to generate light alkanes, i.e., ethane, propane, and butane, which can then be dehydrogenated into the corresponding olefins and H_2_ by commercial technologies.

To identify a catalyst with the aforementioned properties and reactivity, the solvent-free hydrogenolysis of *n*-tetracosane (*n*-C_24_H_50_), an oligomer of PE, was first investigated in a batch reactor, as discussed in detail in the Supporting Information. Among the different bulk metal oxides screened, cobalt oxide (Co_3_O_4_) was found to be highly active, fully converting the paraffin substrate into almost exclusively CH_4_ (Table S1). Given these results, Co_3_O_4_ was tested for the batch solvent-free hydrogenolysis of PE and PP with mass average molecular weights (*M*_W_) of 4000 Da and 12 000 Da, respectively (Figures S1 and S2). After 20 h at 523 K and 40 bar of H_2_, both polymers could be fully converted into CH_4_ over 100 mg of Co_3_O_4_. The dominant products across temperatures, reaction times, and catalyst loadings tested over Co_3_O_4_ were solids or gases, with gaseous products composed exclusively of CH_4_. Under all conditions investigated, only trace liquid products were formed (Figures S1 and S2). These observations support the hypothesis that Co_3_O_4_ favors a terminal C–C bond cleavage mechanism.

Support interactions have been shown to strongly affect the activity and selectivity of C–C bond cleavage over cobalt-based systems in different reactions.^32−36^ Thus, we dispersed 5 wt % cobalt over various supports, i.e., amorphous silica–alumina (SIRAL), silica (SiO_2_), ceria (CeO_2_), zirconia (ZrO_2_), titania (TiO_2_; anatase phase), and ZSM-5 zeolite (Si/Al = 11.5) via incipient wetness impregnation. The catalysts were characterized by temperature-programmed reduction with H_2_ (H_2_-TPR), exhibiting at least two peaks at ca. 533 and 603 K, similar to bulk Co_3_O_4_ (Figure S3), which are characteristic of Co^3+^ and Co^2+^ reduction, respectively.^37^ Notable exceptions to this trend were Co/SIRAL and Co/ZSM-5, both showing a single peak at 533 and 568 K, respectively. The catalysts were then tested in the batch solvent-free hydrogenolysis of model PE (*M*_W_ = 4000 Da) using an equivalent mass of cobalt across the experiments (Figure 2), where *W*_M_ represents the mass of Co metal. The catalytic activity was measured by quantifying the H_2_ conversion, *X*_H_2__, which provides an estimate of the numbers of C–C bonds cleaved. After 20 h at 523 K and 40 bar H_2_, differences were observed in the catalyst performance. In summary, the catalytic activity increased as Co/SIRAL < Co/SiO_2_ < Co/CeO_2_ < Co/ZrO_2_ < Co/TiO_2_ ≪ Co/ZSM-5 (Figure 2a). The reactivity hierarchy was well reflected by the phase distribution of products, with Co/SIRAL, Co/SiO_2_, Co/CeO_2_, Co/ZrO_2_, and Co/TiO_2_ predominantly resulting in solids (85–90%), while Co/ZSM-5 mainly yielded gaseous products (87%). Still, the H_2_ conversion over Co/ZSM-5 was significantly lower than that obtained over Co_3_O_4_ under equivalent conditions (30% vs 60%).

**Figure 2:** Mass-based (a) phase distribution of products and molar H_2_ conversion and (b) gas composition at ca. 5 mol % H_2_ conversion in the hydrogenolysis of PE over the supported cobalt-based catalysts. (c) Gas-phase composition as a function of time in the hydrogenolysis of PE over Co/ZSM-5. The corresponding mass-based phase distribution and molar H_2_ conversion are shown in Figure S5. Conditions: (a–c) *T* = 523 K, *P* = 40 bar H_2_, *W*_M_ = 50 mg; (a) τ = 20 h; (b, c) τ = 5–80 h.

The weight-based selectivity distributions in the gas phase (eq 3 in the SI) were compared at *X*_H_2__ ≈ 5% (Figure 2b), obtained by varying the reaction time. This allows for a more direct performance comparison at an approximately equal number of C–C bonds cleaved. Co/ZrO_2_ exhibited a gas-phase composition virtually comparable to that of bulk Co_3_O_4_. Co/TiO_2_, Co/SiO_2_, Co/CeO_2_, and Co/SIRAL conversely exhibited an increased formation of light alkanes, ranging from C_2_H_6_ to C_5_H_12_, although CH_4_ remained the dominant product (Figure 2b). Interestingly, at reduced H_2_ conversions (≤1%) as obtained after 20 h, a considerably higher fraction of C_3_H_8_ and other light alkanes (60–90 wt %) were detected over Co/SiO_2_ and especially Co/SIRAL (Figure S4). However, the total gas yield was limited to approximately 15%, and by increasing the H_2_ conversion, the amount of CH_4_ rose quickly at the expense of other alkanes (Figure 2b). Notably, Co/ZSM-5 was the only system that did not produce CH_4_ and instead favored the generation of C_3_H_8_ (77%), C_2_H_6_ (12%), and C_4_H_10_ (8%) at *X*_H_2__ ≈ 5% (Figure S5). Under these conditions, almost 30% of the products comprised liquid hydrocarbons (primarily C_5_) with an iso/normal paraffin ratio of ca. 5:1, while higher alkanes were significantly less abundant (Figure S5). The liquid distribution observed for Co/ZSM-5 strongly differs from that obtained over archetypical Ru/C that peaks at around C_16_H_34_.^20^ On the contrary, it qualitatively resembled that obtained over other cobalt-based catalysts, i.e., Co/SiO_2_, Co/CeO_2_, and Co/SIRAL (Figure S6), although these systems generated considerably less liquids (<5 wt %). These results also significantly differ from reports of the hydropyrolysis and hydrocracking of PE over cobalt-based catalysts including CoAl_2_O_4_ and Co/MOR at temperatures ranging from 623 to 823 K, which produce gasoline-range hydrocarbons.^38,39^

The batch hydrogenolysis of *n*-tetracosane was also investigated over Co/ZSM-5. After 2 h, around 70% of C_24_H_50_ and 10% of H_2_ were converted into an almost equal mass mixture of gases, liquids, and solids, resembling the product distribution obtained after 5 h in PE hydrogenolysis at similar (8%) H_2_ conversion (Figures S5 and S7). Notably, the gas phase was predominantly composed of propane (76%), and the distribution of liquids also resembled that obtained after 5 h in PE hydrogenolysis, demonstrating the replicability of our results in a model system.

To probe catalyst stability, we performed a recycling experiment of PE (*M*_W_ = 4000) hydrogenolysis over Co/ZSM-5. The spent catalyst from hydrogenolysis (20 h, 523 K, 40 bar H_2_) was extracted, washed with cyclohexane, dried at 393 K for 12 h, and then reloaded in the Parr reactor with fresh polymer and run under the same reaction conditions. The recycled catalyst exhibited minimal change in activity, maintaining propane as the major gaseous product with only a slight decrease in *X*_H_2__ (Figure S8). To further demonstrate the stability of the Co/ZSM-5 system, we also ran vapor-phase hydrogenolysis of *n*-dodecane in continuous flow, which maintained stable activity and selectivity for at least 24 h on stream (Figure S9a,b). We estimated this system to have a turnover number (TON) of at least 2000 under these conditions. This value fits the criteria of Kozuch and Martin, which state that an industrially relevant catalyst should have a TON ≥1000.^40^

By progressively varying the reaction time from 5 to 80 h, the H_2_ conversion over Co/ZSM-5 increased from ca. 7% to 42% along with the gas fraction (up to ca. 94%) (Figure 2c and Figure S5). Additionally, CH_4_ weight-based selectivity in the gas phase rose with reaction time from 1% to 12% at the expense of C_3_H_8_ production, suggesting that CH_4_ formation is kinetically limited. The cobalt-based catalysts were also tested in the batch solvent-free hydrogenolysis of model PP (*M*_W_ = 12 000 Da) (Figure S10). A comparable activity hierarchy to that in PE hydrogenolysis was observed when deconstructing PP: Co/SIRAL < Co/SiO_2_ < Co/CeO_2_ < Co/ZrO_2_ < Co/TiO_2_ ≪ Co/ZSM-5. Contrastingly, the H_2_ conversions were lower, and the fraction of solids was higher when compared to those obtained for PE hydrogenolysis over the same systems, in agreement with the previous results on Co_3_O_4_ (Figure S10). However, a similar product distribution to that in PE hydrogenolysis was observed, with Co/ZSM-5 favoring C_3_H_8_ formation (ca. 80%), while other systems preferably yielded CH_4_.

Co/ZSM-5, Co/SiO_2_, Co/SIRAL, and the corresponding bare supports, were further characterized by temperature-programmed desorption of NH_3_ (Figure S11). While Co/SiO_2_ is not acidic, Co/ZSM-5 and Co/SIRAL showed two similar main peaks for NH_3_ desorption (423 K, 778 K vs 393 K, 723 K), indicating qualitatively similar acidic strength, although differing in total quantity of sites (0.87 mmol NH_3_ g_cat_^–1^ vs 0.04 μmol NH_3_ g_cat_^–1^, respectively). No differences were observed between the NH_3_-TPD profiles of the metal-containing catalysts and the bare supports, with the exception of a 100 K upward shift of the high-temperature desorption peak in Co/ZSM-5 and of a new peak at 723 K over Co/SIRAL, which might be related to the ability of cobalt to coordinate with NH_3_.^41^ These results, in combination with the analysis of *iso*/normal alkane distribution in the liquid phase during PE hydrogenolysis, provide important mechanistic insights. Specifically, over nonacidic catalysts, such as Co/SiO_2_, normal C_5+_ alkanes were the only liquid products detected in PE hydrogenolysis. In contrast, systems with acid supports like SIRAL and ZSM-5 generated a distribution of *iso*- and *n*-alkanes in the liquid phase (Figure S6). After 5 h of PE hydrogenolysis, Co/ZSM-5 generated primarily C_5+_*iso*-alkanes, indicating the occurrence of isomerization. Accordingly, tertiary carbon could be formed even in the case of PE,^42^ which would explain the similar product distribution observed for PP. These insights point to a possible bifunctional hydrocracking mechanism, also known as ideal hydrocracking,^43^ where both metal-based phases and acid sites are involved.

Co/ZSM-5 was further analyzed by transmission electron microscopy (TEM) prior to and after PE hydrogenolysis. The average particle diameters before and after reaction were 1.50 ± 0.32 and 1.66 ± 0.40 nm, respectively, demonstrating minimal change in particle size (Figure 3a,b and Figures S12 and S13). The minor decrease in activity exhibited by the recycled catalyst (Figure S8) could be due to the slight sintering of nanoparticles after the reaction. The choice of the support has been shown to significantly influence the oxidation state of cobalt, allowing the stabilization of either metallic or partially reduced phases in H_2_-rich atmospheres.^44^ It has been shown that metal confinement within zeolites can stabilize metastable phases,^45−47^ which could offer a possible explanation for the pronounced stabilization effect with ZSM-5. Interestingly, Have et al. demonstrated that H_2_ activation routes differ depending on the cobalt oxidation state in CO_2_-based Fischer–Tropsch synthesis. In particular, they showed that while H_2_ is adsorbed dissociatively over metallic cobalt, cobalt oxide follows a H_2_-assisted pathway.^48^ In addition to the potential influence of acidity as previously discussed, the observed shift from mainly terminal to close-to-terminal C–C bond cleavage in polyolefin hydrogenolysis over Co/ZSM-5 might stem from the preferential stabilization of oxidized cobalt phases by the zeolite that are different from those observed for bulk Co_3_O_4_ or other supports under reductive conditions.

**Figure 3:** Transmission electron microscopy images of Co/ZSM-5 (a) prior to and (b) after PE hydrogenolysis. (c) Temperature-programmed reaction with H_2_ and (d) experimental FT-EXAFS spectra at the Co K-edge of Co/ZSM-5 and Co_3_O_4_ prior to (fresh, black) and after PE hydrogenolysis (used, red). Fits with imaginary components are plotted for fresh (gray, blue, and green lines) and used (pink, orange, and yellow lines) Co/ZSM-5 and were performed using a *k* range of 2.0–10.0 Å^–1^ and an *R* range of 1.0–2.1 Å. Conditions: *T* = 523 K, *P* = 40 bar H_2_, *W*_M_ = 50 mg, τ = 20 h.

To test this hypothesis, we conducted *ex situ* H_2_-TPR as well as X-ray absorption spectroscopy (XAS) at the Co K-edge of Co/ZSM-5 and Co_3_O_4_ after PE hydrogenolysis and compared it to the corresponding data in fresh form (Figure 3c,d and Figure S14). Analysis of the X-ray absorption near-edge structure (XANES) revealed that, while fresh Co_3_O_4_ featured the expected mixed Co^2+^ and Co^3+^ oxidation states, the white line and edge position of the Co/ZSM-5 spectrum resemble those of highly dispersed Co^2+^ species (Figure S14).^49,50^ Notably, the H_2_-TPR profile of the spent Co/ZSM-5 showed new peaks at 603 and 828 K (Figure 3c), indicating the presence of species that are less reducible. These data are consistent with the XANES profiles of spent Co/ZSM-5 showing the preservation of Co^2+^ species, as well with the FT-EXAFS analysis that showed unchanged local coordination environments after reaction, with the first peak centered at 1.61 Å that can be assigned to Co–O by EXAFS analysis (Figures S14–S16 and Table S2). Still, XAS cannot clearly differentiate between Co–O bonds of oxides and Co–C bonds of carbides or oxycarbides, which might form under the reaction conditions studied here. During continuous-flow *n*-dodecane hydrogenolysis, a 4 h induction period was observed where conversion increased from ca. 30% to 46%, and CH_4_ production leveled down from 12% to 2% (Figure S9b). These results suggest that the state of the catalyst is evolving during hydrogenolysis, possibly forming carbide-like species that can be stabilized in MFI frameworks under hydrocarbon-rich reductive environments and that have been shown in Fischer–Tropsch synthesis to be active and to reduce CH_4_ formation.^51,52^ Furthermore, differences in intensity and broadening of the pre-edge XANES region were observed between the spectra of fresh and used Co/ZSM-5 (Figure S17), suggesting changes in the coordination geometry,^53−55^ which could be related to catalyst evolution. Contrarily, there was extensive reduction of the Co_3_O_4_ during PE hydrogenolysis, as observed by a >100 K downward shift in the maxima of the H_2_-TPR profile and an order of magnitude lower H_2_ consumption (Figure 3c) as well as by XAS, which detected almost exclusively metallic cobalt species with the main peak centered at 2.15 Å (not phase corrected) ascribed to Co–Co pairs (Figure 3d and Figures S14–S18). Finally, TEM and XAS were also conducted on Co/SiO_2_ prior to and after PE hydrogenolysis. These analyses revealed that this catalyst was composed of large clusters (*d*_p_ ≈ 17 nm) of Co_3_O_4_ that reduced to CoO-like species upon reaction (Figures S15–S17, S19, and S20). These results suggest that the stabilization of highly dispersed oxidic cobalt nanoparticles by the zeolite prevents complete reduction to metallic species and/or formation of large clusters, which may be related to the observed promotion of C_3_H_8_ and suppression of CH_4_. These results exemplify the complexity of this reaction network, which calls for dedicated and systematic full studies that can properly deconvolute acid- from metal-based bond activation, as well as mass transport and confinement effects, among others.

Thermogravimetric analysis (TGA) of Co/ZSM-5 and Co/SiO_2_ was conducted prior to and after PE hydrogenolysis to probe the presence of coke, since the latter is not directly observable by TEM and XAS. No differences were observed between the TGA curves of fresh and used Co/ZSM-5, indicating the absence of any carbonaceous residues (Figure S21a). Conversely, almost 50% weight loss was observed in the profile of spent Co/SiO_2_ (Figure S21b), which was attributed mainly to the catalyst being coated by solid long chain alkanes rather than coke, as they were the main product obtained over this system (Figure 2a).

ZSM-5-supported cobalt catalysts with different metal loadings (10, 15, and 20 wt %) were further synthesized via incipient wetness impregnation and compared against 5 wt % Co/ZSM-5 in PE hydrogenolysis at equivalent temperature, pressure, time, and cobalt loading (Figure 4a). In particular, while H_2_ conversion remained similar over both Co/ZSM-5 and 10-Co/ZSM-5 (∼29%), it increased over 15-Co/ZSM-5 (32%) and further over 20-Co/ZSM-5 (38%). While the gas fraction remained roughly constant over the catalysts at ca. 87%, differences were observed in the remaining products. Solids were the main byproducts over Co/ZSM-5 and 10-Co/ZSM-5, while liquids, primarily composed of pentane, were observed over 15-Co/ZSM-5 and 20-Co/ZSM-5. However, the most striking difference was found in the composition of the gaseous components; namely, while Co/ZSM-5 and 10-Co/ZSM-5 maintained high weight-based selectivity in the gas phase toward C_3_H_8_ (∼84%), this value decreased over 15-Co/ZSM-5 (66%) and especially 20-Co/ZSM-5 (47%) at the benefit of CH_4_ (14% vs 36%) (Figure S22).

**Figure 4:** Mass-based (a) phase distribution of products and molar H_2_ conversion and (b) CH_4_ and C_3_H_8_ weight-based selectivity in the gas phase as a function of average particle size, *d*_p_, in the hydrogenolysis of PE over ZSM-5-supported cobalt-based catalysts with different metal loadings. Conditions: *T* = 523 K, *P* = 40 bar H_2_, *W*_M_ = 50 mg, τ = 20 h. (c) Phase distribution of products and molar H_2_ conversion over ZSM-5 with loadings corresponding to the equivalent ZSM-5 content in the series presented in panel a).

To gain insights into this phenomenon, we performed TEM and H_2_-TPR of these systems in fresh form. The micrographs of 10-Co/ZSM-5 evidenced well-dispersed particles with a relatively narrow particle size distribution centered around 2.22 ± 0.46 nm (Figure S23), which agreed well with TEM measurements of similarly synthesized 10-Co/ZSM-5 from the literature.^56^ The H_2_-TPR profile of 10-Co/ZSM-5 showed a main peak at 578 K, comparable to Co/ZSM-5 (5 wt %), with a small shoulder at 533 K, accounting for only 5% of the total H_2_ consumption (Figure S24). The similar morphology and reducibility of the 5 and 10 wt % loaded systems are consistent with their analogous catalytic performance. Conversely, 15-Co/ZSM-5 and particularly 20-Co/ZSM-5 showed large ∼30 nm clusters deposited on the external surface of the zeolite together with small nanoparticles dispersed in the microporous structure (Figures S25 and S26), resulting in broad particle size distributions of 4.67 ± 3.30 nm over 15-Co/ZSM-5 and 8.01 ± 5.32 nm over 20-Co/ZSM-5. Their H_2_-TPR profiles exhibited a main peak at 578 K, similar to those observed over Co/ZSM-5 and 10-Co/ZSM-5 that were attributed to the presence of small nanoparticles stabilized by the zeolite, as well as shoulders at 533 and 603 K likely associated with large clusters of Co_3_O_4_ (Figure S24). The area of the combined shoulders represented over 15% and 30% of the total H_2_ consumption of 15-Co/ZSM-5 and 20-Co/ZSM-5, respectively, which would explain both the increased reactivity and the shift toward CH_4_ formation. The dependency of the C_3_H_8_ and CH_4_ weight-based selectivity in the gas phase on the average particle size, *d*_p_, is depicted in Figure 4b. The generation of C_3_H_8_ and CH_4_ followed a volcano and antivolcano behavior with a maximum at 84% and minimum at 1%, respectively, both centered around 2.22 nm obtained over 10-Co/ZSM-5.

While the ZSM-5 modifies the activity of the cobalt oxide, the zeolite itself is also active for propane formation from PE under these conditions. To ensure that observed trends in Figure 4a,b were not a function of the loading of ZSM-5,which decreases as the cobalt loading increases, the activities over equivalent masses of ZSM-5 for the series were measured for PE hydrogenolysis. The results, shown in Figure 4c and Figure S22b, indicate that ZSM-5 alone has high activity for propane formation, although the product selectivity and trends differ in a number of ways. First, the total quantities of gas and liquid produced, as well selectivity to methane, generally increase with increasing loading of ZSM-5, as opposed to Figure 4b which shows a maximum of propane selectivity at an intermediate cobalt loading. This confirms that the selectivity trends in Figure 4b are not an artifact of the decreasing ZSM-5 content with increasing cobalt loading. Second, the liquid products differ between Co/ZSM-5 and ZSM-5. The liquid products over ZSM-5 are largely aromatic and unsaturated hydrocarbons, as evidenced by GC-MS (Figure S27) and by the yellow color of the products (Figure S28), whereas the liquid products over Co/ZSM-5 also contain saturated hydrocarbons and are translucent in color (Figures S27 and S28). This suggests that the cobalt facilitates H_2_ activation to saturate hydrocarbons. Third, unlike the reaction over Co/ZSM-5, in which *X*_H_2__ increases with increasing gas and liquid produced, the *X*_H_2__ over ZSM-5 remains fairly constant. This suggests that there is hydrogen going toward C–C bond cleavage that comes not only from the molecular H_2_ supplied but also from the substrate itself. The evidence of aromatic products is consistent with the theory that hydrogen transfer reactions from the PE substrate are occurring over ZSM-5.

To further probe the role of hydrogen transfer reactions, control reactions of PE (*M*_W_ = 4000) over 5-Co/ZSM-5 and ZSM-5 were performed in a nitrogen atmosphere at 523 K (Figures S29 and S30). In N_2_, both reactions produced gaseous and liquid products, largely composed of light hydrocarbons and a mixture of aromatics. TGA of the ZSM-5 before and after reaction in H_2_ (Figure S21c) revealed a small additional weight loss feature, which could be attributed to soft coke, that is not present over used 5-Co/ZSM-5. In a nitrogen atmosphere, both 5-Co/ZSM-5 and ZSM-5 exhibited coking after reaction (Figure S21d,e). The stability of the ZSM-5 was also tested in a flow reactor for the vapor-phase hydrogenolysis of *n*-dodecane at 523 K over 24 h on stream (Figure S9c,d), exhibiting a slight deactivation over time, which could be due to the soft coke formation in the absence of cobalt.

The most selective bifunctional catalyst, 10-Co/ZSM-5, was selected for testing the solvent-free hydrogenolysis of polyolefins representative of plastic waste: low-density PE (LDPE), PP (*M*_W_ = 12 000 Da), a weight-equivalent mixture of LDPE and PP, as well as a postconsumer PE bottle (post-PE) from VWR International (Figure 5), as described in the Supporting Information. High H_2_ conversion (*X*_H_2__ ≥ 35%) was reached in LDPE and post-PE hydrogenolysis over 10-Co/ZSM-5, leading to gases (ca. 95%). On the contrary, *X*_H_2__ decreased to 25% and 18% in the hydrogenolysis of the LDPE+PP mixture and PP, resulting in a higher solid fraction (ca. 30% and 60%), respectively, compared to LDPE alone and post-PE (<3%; Figure 5a), probably due to the lower reactivity of PP. In all cases, liquids were limited to ≤5 wt % and were composed primarily of C_5_ (Figure S31), as observed in PE hydrogenolysis over Co/ZSM-5. C_3_H_8_ was preferably formed in all tests, reaching ca. 80% weight-based selectivity in the gas phase (Figure 5b). Together with the tests on *n*-C_24_H_50_ hydrogenolysis, these results showcase that the favored propane formation in the gas phase can be obtained over a wide range of substrates.

**Figure 5:** Mass-based (a) phase distribution of products and molar H_2_ conversion and (b) gas composition in the hydrogenolysis of LDPE, PP, LDPE+PP, and post-PE over 10-Co/ZSM-5. Conditions: *T* = 523 K, *P* = 40 bar H_2_ (35 bar H_2_ for post-PE), *W*_M_ = 50 mg, τ = 40 h (50 h for post-PE).

Finally, we examined the effect of different zeolite topologies on the catalytic activity and selectivity for PE depolymerization. Catalysts containing 5 wt % Co were synthesized via incipient wetness impregnation using three additional zeolite supports: FAU (Si/Al = 15), BEA (Si/Al = 12.5), and MOR (Si/Al = 10). Catalyst characterizations for these materials, including XRD, H_2_-TPR, and NH_3_-TPD, are shown in Figure S32, which confirms that the materials are crystalline and that the cobalt oxide domains have relatively similar reducibility. PE reactions were carried out at 523 K, under 40 bar H_2_, over 20 h (Figure 6). As shown in Figure 6a, catalyst activity varies significantly, with *X*_H_2__ increasing from Co/MOR < Co/BEA < Co/FAU < Co/ZSM-5. While Co/FAU, Co/BEA, and Co/MOR produced similar quantities of gas, the liquid composition of Co/FAU and Co/BEA was significantly higher (38% and 51%, respectively) compared to 3% and 4% over ZSM-5 and MOR, respectively. The liquid product distributions (comprising C_8_–C_18_ saturated and unsaturated hydrocarbons) are shown in Figure S33. Some variations can also be observed in the selectivity within the gas phase (Figure 6b), with cobalt supported on FAU, BEA, and MOR exhibiting slightly higher butane selectivity (up to 18% over FAU and MOR). These results demonstrate the potential to use the zeolite support as a handle to tune product distributions.

**Figure 6:** Mass-based (a) phase distribution of products and molar H_2_ conversion and (b) gas composition in the hydrogenolysis of PE over different zeolite-supported cobalt-based catalysts. Conditions: *T* = 523 K, *P* = 40 bar H_2_, *W*_M_ = 50 mg, τ = 20 h.

In conclusion, we demonstrated ZSM-5-supported cobalt-based catalysts as highly efficient systems for the selective conversion of PE and PP into C_3_H_8_ (up to 84%), with a balance of other light alkanes including C_2_H_6_ and C_4_H_10_. By applying commercial dehydrogenation technologies, these alkanes could be readily converted into the corresponding olefins and H_2_, closing both the carbon and hydrogen loop in the production and regeneration cycle of these polyolefins. The performance of Co/ZSM-5 significantly differed from that of bulk Co_3_O_4_ as well as those of other cobalt-based systems supported on other carriers, which led to the almost exclusive formation of CH_4_ (up to 95%). The ability to shift from terminal C–C bond cleavage to cleavage at regular intervals in the internal polymer backbone was ascribed to the stabilization of dispersed oxidic cobalt nanoparticles and the ZSM-5 support itself. Further, the cobalt loading was varied, which revealed a volcano and antivolcano behavior of the C_3_H_8_ and CH_4_ weight-based selectivity in the gas phase with the particle size, respectively. In particular, C_3_H_8_ production peaked at 2.22 nm over 10-Co/ZSM-5, while it decreased until ca. 30% over 20-Co/ZSM-5 at the benefit of CH_4_. This behavior was ascribed to the progressive accumulation of large Co_3_O_4_ clusters (up to 30 nm) with cobalt loading on the external zeolite surface. After optimizing the metal loading, we demonstrate that 10 wt % Co/ZSM-5 can selectively catalyze the solvent-free hydrogenolysis of low-density PE (LDPE), mixtures of LDPE and PP, as well as postconsumer PE. Finally, we demonstrated that the choice of zeolite support can influence product distributions and activity, providing opportunities to increase liquid yields and shift propane/butane selectivity in the gas phase.

While these results show promise, there are many remaining open questions, including the influence of zeolite acidity, and the role that topology, porosity, and confinement play in determining activity and product distributions. In addition, process design considerations including reactor selection, technoeconomic analysis, life cycle assessment, and the influence of relevant contaminants and additives on reactivity will be critical to develop viable technologies for polyolefin upcycling.

## Experimental Section

### Catalyst Synthesis and Characterization

Commercial oxides, such as Co_3_O_4_, were calcined at 673 K for 5 h prior to their use in the catalytic tests. Commercial supports, i.e., SiO_2_, CeO_2_, ZrO_2_, TiO_2_, and SIRAL-40, as well as ZSM-5, FAU, BEA, and MOR zeolites, were calcined at 823 K for 5 h prior to their use as carriers in the catalyst preparation. Supported cobalt-based catalysts were prepared by incipient wetness impregnation. The metal precursor Co(NO_3_)_2_·6H_2_O was dissolved in a volume of deionized water equal to the pore volume of the carrier in appropriate amounts to achieve the desired loading (5, 10, 15, or 20 wt %) calculated on a metal basis. After drying at 423 K for 2 h, the samples were calcined at 673 K for 5 h prior to their use in the catalytic tests. The catalysts are referred to as ω_metal_-Co/*C*, where *C* represents the carrier, i.e., SiO_2_, CeO_2_, ZrO_2_, TiO_2_, SIRAL, or ZSM-5, and ω_metal_ defines the weight percentage of metal, which is omitted for the materials with 5 wt % loading. The crystalline order, redox and acidic properties, particle dispersion, cobalt oxidation state, and the presence of coke in the fresh and/or used catalysts were characterized using powder X-ray diffraction, temperature-programmed reduction with H_2_, temperature-programmed desorption of NH_3_, transmission electron microscopy, X-ray absorption spectroscopy, and thermogravimetric analysis, respectively. Full details are provided in the Supporting Information.

### Catalyst Testing

The catalytic tests were performed in a 25 cm^3^ stainless steel Parr reactor setup. Briefly, the solid alkanes (weight, *W* = 0.7 g)—*n*-C_24_H_50_, polyethylene (PE, mass average molecular weight, *M*_w_, 4000 Da), polypropylene (PP, *M*_w_ = 12 000 Da), low-density PE (LDPE; melt flow index, MFI, 25 g in 10 min at 463 K and 2.16 kg), and postconsumer LDPE (post-LDPE)—were loaded in the reactor together with the catalyst in an appropriate amount to ensure that, across different catalytic tests, the same amount of Co metal was used (mass metal equivalent, *W*_M_ = 25–100 mg). The reactor was then evacuated, flushed, and pressurized (*P* = 40 bar) with H_2_. The reactor was then placed in a homemade heater equipped with a Digi-Sense TC9100 temperature controller and a K-type thermocouple to regulate the operating temperature (*T* = 523 K), insulated, and run for different reaction times (τ = 5–80 h). After the tests, the reactor was quenched in an ice bath. The gaseous alkane products and H_2_ in the headspace were collected in a gas sampling bag and were quantified off-line using a gas chromatograph (GC) coupled to a flame ionization detector (FID) and a thermal conductivity detector. Liquid alkane products (C_5_–C_32_) were extracted from the remaining solid alkanes (C_32+_) and catalyst using cyclohexane or acetone as solvent. Then, 1,3,5-tritertbutyl benzene was added as an external standard, and the suspension was centrifuged to separate liquids and solids. The liquid products were identified using GC coupled to a mass spectrometer and then quantified off-line using a GC-FID. The solids were then dried overnight and weighted. After the products were extracted, the catalyst was retrieved for further characterization. The catalyst activity in the hydrogenolysis of polyolefins was measured based on the number of C–C bonds cleaved, which was estimated from the conversion of H_2_. The phase-based selectivity (solid, liquid, gas) was determined by dividing the measured mass of product in a given phase by the total mass of product quantified, while the weight-based product selectivities in the gas phase were estimated by the ratio of the mass of a given gaseous product and the total mass of gaseous products. Full details are provided in the Supporting Information.

## Supporting Information Available

Catalyst synthesis, reactivity testing, additional figures, and data of further catalytic experiments and catalyst characterization (PDF)
